# Effects of Warm Needle Acupuncture plus Xitong Waixi Lotion in Patients with Knee Osteoarthritis: A Randomized Controlled Trial

**DOI:** 10.1155/2022/5467712

**Published:** 2022-08-04

**Authors:** Guanyun Sheng, Jing Yang, Peng Rong, Xueyi Yang

**Affiliations:** ^1^Department of Orthopaedics, Liuzhou Traditional Chinese Medical Hospital, Guangxi University of Chinese Medicine, Liuzhou 545001, China; ^2^Intensive Care Unit, Liuzhou Traditional Chinese Medical Hospital, Guangxi University of Chinese Medicine, Liuzhou 545001, China; ^3^Graduate School, Guangxi University of Chinese Medicine, Nanning 530000, China

## Abstract

**Objective:**

To evaluate the effect of warm needle acupuncture plus Xitong Waixi lotion on the levels of IL-1, TNF-*α*, and MMP-3 in patients with knee osteoarthritis.

**Methods:**

Eighty patients with knee osteoarthritis admitted to our hospital from October 2019 to June 2021 were recruited and assigned via the random number table method at a ratio of 1 : 1 to receive either Xitong Waixi lotion (conventional group) or warm needle acupuncture plus Xitong Waixi lotion (combined group). Outcome measures included clinical efficacy, inflammatory cytokine level, Western Ontario and McMaster Universities Arthritis Index (WOMAC) score, visual analogue scale (VAS) score, Hospital for Special Surgery (HSS) knee score, and adverse reactions.

**Results:**

Warm needle acupuncture plus Xitong Waixi lotion was associated with a significantly higher clinical efficacy versus Xitong Waixi lotion alone (*P*=0.006). Patients in the combined group had significantly lower levels of interleukin (IL)-1, tumor necrosis factor-*α* (TNF-*α*), and matrix metalloproteinase-3 (MMP-3) than those in the conventional group (*P*=0.020). Warm needle acupuncture plus Xitong Waixi lotion resulted in significantly lower WOMAC scores and VAS scores and higher HSS scores for the patients versus Xitong Waixi lotion (*P*=0.012). The two groups had a similar incidence of adverse events (*P*=0.068).

**Conclusion:**

Warm needle acupuncture plus Xitong Waixi lotion effectively alleviates the inflammatory response and knee pain in patients with knee osteoarthritis, with significant clinical effects and a high safety profile.

## 1. Introduction

Osteoarthritis of the knee joint is a common and clinically prevalent disease in the middle-aged and elderly population [1]. Osteoarthritis of the knee is caused mainly by the deformity of the joint due to osteophytes and changes in the articular cartilage, which impairs the joint function of the knee [2]. In recent years, the incidence of osteoarthritis of the knee has been on the rise [3]. Clinical studies have shown that the inflammatory cytokines interleukin-1 (IL-1), tumor necrosis factor-alpha (TNF-*α*), and matrix metalloproteinase-3 (MMP-3) are closely associated with the development of osteoarthritis of the knee [3]. During the development of osteoarthritis of the knee, IL-1 and TNF-*α* stimulate the synovium to promote the production and secretion of synovial cells and chondrocytes, including inflammatory transmitters such as MMP, which degrade the patient's articular cartilage proteoglycans and collagen and accelerate the production and secretion of synovial cells and chondrocytes disease [1]. In the presence of IL-1 and TNF-*α*, the patient's synovial macrophages further differentiate into osteoclasts, leading to destruction of the marginal bone and inhibition of matrix repair [2]. TNF-*α* also induces the production of other inflammatory factors, and IL-1 increases the activity of TNF-*α*, which can act synergistically to cause articular cartilage tissue damage in patients [4]. MMP-3 is thought to be a key matrix metalloproteinase causing bone destruction in knee osteoarthritis and is a major mediator of knee osteoarthritis damage. It degrades a large number of extracellular matrix components and activates other MMPs in vivo, triggering bone destruction in patients by degrading type II collagen [3]. Fang et al. found that abnormal expression of MMPs directly led to degradation of articular cartilage in patients, resulting in bone destruction and damage [2].

The early symptoms of the disease are relatively mild and are mostly treated with conservative medication; however, the prolongation of the disease and the aggravation of symptoms result in compromised treatment outcomes with conventional drugs [4]. Currently, there is no clinical cure for osteoarthritis of the knee, and clinical treatment primarily aims to relieve patients' symptoms and improve their joint function [5]. Western medicine for patients with osteoarthritis of the knee mostly adopts painkillers, which only temporarily relieve joint pain but are associated with various side effects and are not suitable for long-term use [6]. Prolonged medication in patients with arthritis can not only affect patients' liver and kidney function but also sometimes cause gastrointestinal discomfort such as nausea and vomiting due to the side effects of the drugs. Commonly used nonsteroidal anti-inflammatory drugs (NSAIDs) are the most commonly used drugs to relieve pain and improve joint function in patients with osteoarthritis, including topical drugs and systemically applied drugs [6]. Topical medications are recommended before the use of oral medications, especially in the elderly, with the use of gel patches of various NSAID-based drugs. Topical medications provide rapid and effective relief of mild to moderate pain in joints, and their gastrointestinal adverse effects are mild, but attention needs to be paid to the occurrence of local skin adverse effects [5]. Opioid analgesics can be used for those who are ineffective or intolerant to NSAID therapy, but it is important to note that opioids have a relatively high incidence of adverse reactions and addiction [6]. Joint cavity injections have glucocorticoids, which are mainly anti-inflammatory, but have an effect on cartilage metabolism and should not be used long-term. Joint cavity injections are invasive treatments and may increase the risk of joint infection [7].

In traditional Chinese medicine (TCM), osteoarthritis of the knee joint belongs to the category of “paralysis.” Liver and kidney deficiency leads to deficiency of qi and blood, invasion of cold and dampness in the body, which results in obstruction of meridians and paralysis of qi and blood [7]. Thus, the treatment of patients should focus on tonifying the liver and kidney, dispelling dampness, and relieving pain. The homemade Xitong Waixi lotion of our hospital originated from the “Prescriptions for emergencies,” which is an ancient representative for the treatment of wind-cold-damp paralysis caused by deficiency of liver and kidney and deficiency of qi and blood [8]. In addition, warm needle acupuncture activates qi and blood, warms the meridians, dispels dampness, and relieves pain, which is effective in the treatment of knee osteoarthritis [9]. In the present study, 80 patients with knee osteoarthritis admitted to our hospital from October 2019 to June 2021 were recruited to evaluate the effect of warm needle acupuncture plus Xitong Waixi lotion on the levels of IL-1, TNF-*α*, and MMP-3 in patients with knee osteoarthritis.

## 2. Materials and Methods

### 2.1. Participants

Eighty patients with osteoarthritis of the knee admitted to our hospital from October 2019 to June 2021 were recruited for prospective analysis and allocated to either the conventional group (*n* = 40) or the combined group (*n* = 40) using the random number table method in a 1 : 1 ratio. Study investigators, patients, and data analysts remained blinded until all follow-up data were obtained, and the primary analytic strategies were finalized. The study was reviewed and approved by our medical ethics committee, and all patients themselves and their families were informed and provided written informed consent (approval no.20190366).

### 2.2. Inclusion and Exclusion Criteria

Patients who met the diagnostic criteria of Western medicine and Chinese medicine for osteoarthritis of the knee, aged ≥40 years, and without any recent therapeutic treatment were included.

Patients with other organ systemic diseases, psychiatric diseases, and poor compliance that prevented treatment cooperation were excluded from this study.

### 2.3. Treatment

Patients in the conventional group received Xitong Waixi lotion, and its formula consists of Aconiti Radix Cocta, Radic Aconiti Kusnezoffii Preparata, Herba Asari, safflower, Herba Speranskiae Tuberculatae, Angelicae Pubescentis Radix, Angelicae Sinensis Radix, Paeoniae Radix Rubra, Chuanxiong Rhizoma, Lycopodii Herba, *Kadsura coccinea*, Cyathulae Radix, Clematidis Radix et Rhizoma, Taxilli Herba, Sappan Lignum, Notopterygii Rhizoma et Radix, Dipsaci Radix, olibanum, Myrrha, and Semen Strychni. The above medicinal herbs were decocted with water to obtain 1000 mL of filtrate, and the lotion was used to lave patients' knee joints for 30 min, 2 times daily. A similar regimen of Xitong Waixi lotion was introduced to the patients in the combined group.

Patients in the combined group additionally received warm needle acupuncture. With the patient in a sitting or supine position, the patient's knee joint was kept in flexion at 140°, and a soft cushion was placed under the rouge fossa. Warm needle acupuncture was performed at the acupoints of Dubi, Heding, Zusanli, Yinlingquan, Yanglingquan, and E'shi using 0.35 mm × 60 mm millineedles (Suzhou Acupuncture Supplies Factory) after routine sterilization, and a 1.5 cm moxa stick was placed on the shaft of the needles. The needles were removed after the moxa sticks burned out and the needle handles cooled.

### 2.4. Outcome Measures

1. Western Ontario and McMaster Universities Arthritis Index (WOMAC) score [10]: before and after treatment, the severity of clinical symptoms was assessed in both groups using the WOMAC scale, which included three domains of pain, stiffness, and joint function, with a total of 24 items. Each dimension was scored on a 0–4 points scale. The lower the score, the better the knee function.
2. Clinical efficacy: according to the WOMAC score before and after treatment, the score reduction rate was calculated according to the nimodipine method [11]. Score reduction rate = (integration before treatment − score after treatment) − score before treatment × 100%.
3. Markedly effective: score reduction rate ≥50%, but ≤79%; effective: score reduction rate ≥25%, but ≤49%; ineffective: score reduction rate ≤24%.
4. Inflammatory cytokine levels: 2 mL of joint fluid was collected from both groups of patients before and after treatment and centrifuged to obtain the supernatant, which was stored at −30°C for assay. The levels of interleukin (IL)-1, tumor necrosis factor-*α* (TNF-*α*), and matrix metalloproteinase-3 (MMP-3) of patients were determined by enzyme-linked immunosorbent assay.
5. Visual analogue scale (VAS) score: the VAS was used to evaluate the pain of the knee joint before and after treatment, with a total score of 10 points. The higher the score, the more severe the pain.
6. Hospital for Special Surgery (HSS) scores: the HSS scale was used to evaluate the knee function of patients before and after treatment. The scale consists of six domains, pain, joint function, mobility, muscle strength, knee flexion deformity, and stability, and is scored out of 100 points.
7. Adverse events: adverse events during treatment include nausea, pruritus, skin redness, and swelling

### 2.5. Treatment Methods

SPSS 21.0 was used for data analyses, and GraphPad Prism 8 was used to plot the graph. Measurement data are expressed as (mean ± SD) and analyzed using the independent sample *t*-test, and count data are expressed as cases (%) and analyzed using the chi-square test. Differences were considered statistically significant at *P* < 0.05.

## 3. Results

### 3.1. Baseline Patient Profile

The baseline characteristics of the conventional group (22 males and 18 females, aged 58–77 years, mean age of 65.42 ± 2.28 years, disease duration of 2–7 years, mean disease duration of 3.43 ± 1.21 years, and 32 cases of unilateral lesions and 8 cases of bilateral lesions) were comparable with those of the combined group (25 males and 15 females, aged 59–75 years, mean age of 65.31 ± 2.19 years, disease duration of 1–7 years, mean disease duration of 3.35 ± 1.22 years, and 30 cases of unilateral disease and 10 cases of bilateral disease) (*P* > 0.05) (Table 1).

### 3.2. WOMAC Scores, VAS Scores, and HSS Scores

Warm needle acupuncture plus Xitong Waixi lotion resulted in significantly lower WOMAC scores and VAS scores and higher HSS scores for the patients versus Xitong Waixi lotion (*P* < 0.05) (Figure 1).

### 3.3. Clinical Efficacy

Warm needle acupuncture plus Xitong Waixi lotion was associated with a significantly higher clinical efficacy versus Xitong Waixi lotion alone (*P* < 0.05) (Table 2).

### 3.4. Inflammatory Cytokine Levels

Patients in the combined group had significantly lower levels of IL-1, TNF-*α*, and MMP-3 than those in the conventional group (*P* < 0.05) (Figure 2).

### 3.5. Adverse Events

The two groups had a similar incidence of adverse events (*P* < 0.05) (Table 3).

## 4. Discussion

The knee is a common site of osteoarthritis, and patients with osteoarthritis of the knee usually suffer from a long-term condition that may lead to narrowing of the joint space and fibrotic changes in adjacent tissues, resulting in degenerative changes in the knee cartilage. The quality of life of the joint and the patient is impaired [12]. Patients with osteoarthritis of the knee are commonly treated clinically with western medicine, but a cure has not been achieved, and long-term use of Western medicine has been associated with various adverse effects. The treatment of arthritis patients in Chinese medicine is mainly to activate blood circulation and remove blood stasis [13]. Acupuncture improves microcirculation around the patient's diseased area by stimulating the acupoints, thereby relieving pain and inflammatory responses. Warm needle acupuncture at the Heding, Xuehai, Dubi, and Zusanli acupoints can nourish the qi and blood and dispel cold and dampness to treat osteoarthritis of the knee joint. Blood and qi are concentrated in these acupoints, and acupuncture at these points can unblock the blood vessels around the patient's diseased area to repair the soft tissues of the patient's knee joint, thereby effectively relieving the knee pain [14]. Compared to traditional therapies, acupuncture is highly accepted clinically for its effectiveness in reducing patients' pain and improving knee function with no significant adverse effects [1–17]. Xitong Waixi lotion is commonly used in our hospital to treat patients with arthritis, with a marked effect of dispelling cold and dampness and unblocking the meridians. It allows the medicine to reach the affected area of the patient directly through fumigation, causing the capillaries in the affected area to dilate, thus relieving inflammation and stasis of blood, thus eliminating paralysis and pain [18–23].

In the present study, warm needle acupuncture plus Xitong Waixi lotion was associated with a significantly higher clinical efficacy and better WOMAC scores, VAS scores, and HSS scores versus Xitong Waixi lotion alone, and the two groups had a similar incidence of adverse events, indicating that warm needle acupuncture plus Xitong Waixi lotion is clinically effective in relieving the knee pain with a high safety profile. The reason may be that warm needle acupuncture can quickly repair the diseased tissues of the patient's knee joint to relieve the knee pain, and Xitong Waixi lotion can effectively accelerate the metabolism of the patient's body to reduce the bruising and inflammation of the affected area. A synergistic effect can be achieved by the combination of the two treatment methods [24–27]. Here, patients in the combined group had significantly lower levels of IL-1, TNF-*α*, and MMP-3 than those in the conventional group, suggesting that warm needle acupuncture plus Xitong Waixi lotion can effectively reduce the levels of IL-1, TNF-*α*, and MMP-3 in patients with knee osteoarthritis. The reason may be that the stimulation of the relevant acupuncture points in the warm needle acupuncture treatment resulted in the release of cytokines that inhibit the inflammatory response of the organism, thereby suppressing the production of inflammatory cytokines. However, further clinical studies are required to confirm this conclusion.

By regulating the functions of the human body, TCM can unblock blood vessels and nourish blood and qi (breath power), which are beneficial in improving the immunity of the body [28]. In addition, the clinical efficacy of TCM in treating chronic diseases is remarkable and cost-effective [29]. For instance, in diabetes mellitus, TCM can effectively alleviate the disease by adjusting the patient's diet [30], facilitate the rehabilitation of hemiplegia, arthritis, and lumbar disc herniation, and improve the quality of life of patients using acupuncture [31]. The advantage of Chinese medicine is to improve the overall state of the human body and to improve the nutritional status of the joints from a macroscopic point of view, for example, through the use of various herbs to relax the tendons and activate blood [32]. Western medicine is more concerned with the principle of pathogenesis. For example, in early osteoarthritis of the knee, the pain caused by inflammation is alleviated; in midstage osteoarthritis of the knee, the cartilage is repaired; in advanced osteoarthritis of the knee, the cartilage is worn away and there is no way to save it, so knee replacement surgery is performed [33]. With the development of the times, there is more and more intermingling of Chinese and Western medicine, for example, many Chinese hospitals now also treat by surgery, and Western doctors also use Chinese medicine to supplement Western treatment. Patients can choose to take oral leflunomide to control the condition [34]. If the condition is mild, Chinese herbal medicines can be taken to treat the condition, such as those that invigorate blood stasis and dispel wind and relieve pain, which can achieve good results [35]. If the patient's condition is more severe, it can also be controlled with herbal scalding or moxibustion [36]. This is what is known as a combination of Chinese and Western medicine.

## 5. Conclusion

To sum up, warm needle acupuncture plus Xitong Waixi lotion effectively alleviates the inflammatory response and knee pain in patients with knee osteoarthritis, with significant clinical effects and a high safety profile. However, there are still limitations to our experiment; first, the small sample size in this study and the applicability of the treatment to all populations remain to be verified. Second, as a homemade medicine, further discoveries on its clinical efficacy are needed if it is to gain acceptance from experts nationally and globally.

## Figures and Tables

**Figure 1:** WOMAC scores, VAS scores, and HSS scores ($\bar{x}\pm s$). ^*∗*^*P*=0.012 < 0.05.

**Figure 2:** Inflammatory cytokine levels ($\bar{x}\pm s$). ^*∗*^*P*=0.020 < 0.05.

**Table 1:** Patient characteristics (*n* (%)).

	Conventional (*n* = 40)	Combined (*n* = 40)
Gender		
Male	22	25
Female	18	15

Mean age (year)	65.42 ± 2.28	65.31 ± 2.19

Mean disease duration (month)	3.43 ± 1.21	3.35 ± 1.22

Diseased parts		
Unilateral lesions	32	30
Bilateral lesions	8	10

**Table 2:** Clinical efficacy (*n* (%)).

	Conventional (*n* = 40)	Combined (*n* = 40)	*x * ^2^	*P*
Markedly effective	11	26		
Effective	18	12		
Ineffective	11	2		
Efficacy (%)	29 (73%)	38 (95%)	7.44	0.006

**Table 3:** Adverse events (*n* (%)).

	Conventional (*n* = 40)	Combined (*n* = 40)	*x * ^2^	*P*
Nausea	0	0		
Pruritis	1	0		
Skin redness and swelling	0	1		
Incidence (%)	1 (2.5%)	1 (2.5%)	—	0.068

## Data Availability

No data were used to support this study.
